RETRACTED

# Silent Myocardial Infarction: A Case Report

**DOI:** 10.7759/cureus.43906

**Published:** 2023-08-22

**Authors:** Maria V Kolesova, Suzanne Minor

**Affiliations:** 1 Medical School, Florida International University, Herbert Wertheim College of Medicine, Miami, USA; 2 Office of Academic Affairs, Florida International University, Miami, USA

**Keywords:** myocardial infarction, silent myocardial infarction, old myocardial infarction, electrocardiogram (ecg/ekg), cardiovascular disease prevention, cardiovascular disease risk, cardiovascular disease (cvd), cad: coronary artery disease

## Abstract

Silent myocardial infarction (SMI) is a type of myocardial infarction (MI) that is asymptomatic or demonstrates mild symptoms; therefore, patients often do not seek medical treatment. SMI cases are often incidentally detected later by electrocardiogram (ECG).

We present a case of a 59-year-old overweight woman with prediabetes, primary hypertension, and hypercholesterolemia who presented for herpes zoster (HZ) follow-up; she reported having skipped heartbeats and heart rate fluctuations during the review of systems. On further workup, ECG revealed low voltage QRS complexes, flat QRS complexes, flat T waves, and pathological Q waves, suggesting the diagnosis of SMI. Based on the identified risk factors, including high BMI, prediabetes, primary hypertension, hypercholesterolemia, HZ, and newly diagnosed SMI, the patient was advised to continue with lisinopril 20 mg daily, prescribed atorvastatin 80 mg daily, and was educated about maintaining a healthy diet, exercise, and receiving the shingles vaccination. To prevent the possible risks of poor outcomes such as those following MI, stroke, heart failure, arrhythmias, angina, and shortness of breath (SOB), the patient was referred to the cardiologist for a stress test and further treatment plan.

## Introduction

Myocardial infarction (MI), a common cardiovascular disease (CVD) defined as myocardial necrosis due to coronary ischemia, is a leading cause of death worldwide [1]. Typically, patients presenting with MI may exhibit symptoms of chest pain, squeezing chest pressure, and shortness of breath (SOB) at rest or upon minimal exertion. However, patients with silent myocardial infarction (SMI) are asymptomatic or demonstrate mild symptoms such as slight chest discomfort and often do not seek medical treatment for such mild complaints [1]. Mildly symptomatic SMI cases may be detected upon subsequent electrocardiogram (ECG), nuclear stress test, or cardiovascular MRI [1,2]. The incidence of SMIs ranges from 22% to 60% of all myocardial infarctions [1,2]. SMI is associated with an increased risk of heart failure (HF). Qureshi et al. (2018) reported that the incidence of HF per 1,000 patients a year with SMI versus those without MI was 16.2 and 7.8, respectively (p<0.001) [3]. Mortality due to coronary heart disease is higher among patients with SMI as compared to those who had never had MI [hazard ratio (HR): 3.06; 95% confidence interval (CI): 1.88-4.99]; the same applies to all-cause mortality (HR: 1.34; 95% CI: 1.09-1.65) [2]. SMI leads to scar formation and ventricular dysfunction and could be responsible for thrombus, cardiac embolism, and stroke [4].

RETRACTED

Zhang et al. (2016), in a study involving 9,498 patients, revealed that the risk of mortality from SMI is higher in females when compared to males (p=0.089) [2]. Females, when compared to males, have higher pain tolerance and manifest more atypical symptoms of MI, such as nausea, vomiting, diaphoresis, dizziness, SOB, fatigue in days before MI, and pain in atypical locations other than chest, arm, or jaw, which leads to unrecognition or misdiagnoses and subsequent hospital admissions [5]. The one-year mortality rate after MI is higher among females, with an odds ratio of 1.6 [5]. MI that occurs in patients in the age group of 18-65 years is defined as premature [6]. In a systematic review by Dugani et al. (2019), hypercholesterolemia, hypertension, and diabetes mellitus are identified as risk factors for developing premature MI [6]. The Myocardial Infarction Risk Knowledge Database (MIRKB) was developed to identify individuals at risk of MI [7].

We present a case of SMI in a postmenopausal overweight patient with a history of hysterectomy, prediabetes, primary hypertension, and hypercholesterolemia. We describe the etiology of the condition and discuss the tests to assess for coronary artery disease (CAD) and the treatment options for this patient without health insurance.

## Case presentation

A 59-year-old woman with a past medical history of hysterectomy, overweight, prediabetes, primary hypertension, and hypercholesterolemia visited the clinic for a follow-up of a recent herpes zoster (HZ) rash. Three weeks prior, she had been diagnosed with HZ infection upon presentation with a painful rash in the lumbar area extending to the right posterior thigh. She had completed a 10-day course of acyclovir 800 mg daily and presented with a well-healed rash. During the assessment of her chronic health issues at the follow-up visit, she mentioned that she was concerned about "skipped heartbeats," which had been increasingly noticeable, and her pulse had occasionally reached 100 bpm. She stated that an ECG had been done "a long time ago" and that "it was normal." She presented with no chest pain, SOB, or weakness. Her active list of medications included atorvastatin 10 mg, once a day by mouth, and lisinopril 20 mg, once a day by mouth. Apart from her high BMI of 27.9 kg/m^2^, the patient's cardiovascular and pulmonary physical examination was unremarkable; her vitals were as follows: blood pressure (BP): 138/70 mmHg, oxygen saturation (SaO_2_): 99%, pulse: 77 bpm, respiratory rate (RR): 17 breaths per minute, and temperature (T): 97.5 °F (36.4 °C). Her laboratory results from the last visit, including a comprehensive metabolic panel, complete blood count, lipid panel, and urinalysis, were unremarkable, except for a slightly elevated HbA1C of 5.8% (average HbA1C level: <5.7%). The lipid panel was within the normal reference range with cholesterol of 179 mg/dL, LDL of 90 mg/dL, HDL of 70 mg/dL, and triglycerides of 101 mg/dL. An ECG was performed during the visit, which demonstrated a normal pulse rate, regular rhythm, sinus P waves, normal PR and QT intervals, and normal cardiac axis. The QRS complexes were low-voltage since the sum of QRS amplitudes in leads V1, V2, and V3 was less than 30 mV. The ECG demonstrated Q waves in leads V2 and V3, Q waves with an amplitude of more than 2 mV in lead III, Q waves wider than 0.04 seconds in leads II, aVL, V2, V3, and V6, and flat QRS complex and flat T waves in lead aVF (Figure 1).

RETRACTED

**Figure 1:** ECG of the patient The image shows small Q waves in leads V2 and V3, Q waves with an amplitude of 4-5 mV in lead III, flat QRS complexes, and flat T waves in lead aVF Green arrows: Q waves in leads V2 and V3. Red arrows: Q waves with an amplitude of more than 2 mV in lead III. Blue arrows: flat QRS complex in lead aVF. Yellow arrows: flat T waves in lead aVF ECG: electrocardiogram

Based on the patient's medical history of high BMI, prediabetes, primary hypertension, hypercholesterolemia, and HZ, along with her presenting cardiac symptoms, the ECG results suggested an old inferior MI with Q and T wave findings. After reviewing the patient's medical history and ECG results, the diagnosis of SMI was made. The patient was educated about the abnormal ECG and the possibility of an old SMI. She received a cardiology referral and was asked to return to the clinic after 46 weeks for a follow-up visit. Atorvastatin dosage was increased to 80 mg daily. The patient was also counseled on MI symptoms and instructed to call 911 if she experienced chest pain or SOB. Unfortunately, she had no health insurance, and hence she would likely have difficulty getting a cardiovascular consultation.

## Discussion

Our patient's ECG demonstrated several pathological findings: low voltage QRS complexes, flat QRS complexes and flat T waves in lead aVF, and pathological Q waves. The Q waves were considered pathological due to the following findings: Q waves were present in leads V2 and V3; Q waves wider than 0.04 seconds were seen in leads II, aVL, V2, V3, and V6; Q wave amplitude was more than 2 mV in lead III. The ECG had two limitations: low voltage and motion artifacts. The baseline ECG was unavailable, and hence whether the changes were new or old could not be verified. The ECG alone is not sufficient for detecting an old SMI. ECGs are read in correlation with patient history, and our patient’s history was consistent with a high risk for CAD.

RETRACTED

The patient had undergone a hysterectomy at the age of 47 years. Females who undergo hysterectomy with ovarian conservation at the age of 36-50 years are at an increased risk of developing hyperlipidemia, hypertension, obesity, cardiac arrhythmias, and CAD [8]. The risk for CVD is significantly increased in females who undergo a hysterectomy at the age of 50 years or less [9]. This was an unmodifiable risk factor for our patient.

The patient had suffered from chickenpox in childhood, and then the latent varicella zoster virus (VZV) had developed HZ or shingles. HZ in adults can be associated with cerebrovascular and cardiac events, including acute strokes and MI [10]. Kim et al. (2017) revealed that HZ was associated with a 35% increased risk of stroke (HR: 1.35; 95% CI: 1.18-1.54) and a 59% increased risk of MI (HR: 1.59; 95% CI: 1.27-2.01) [11]. Yawn et al. (2016) found that HZ in patients older than 50 years is associated with stroke and MI [12]. Our patient was prescribed acyclovir 800 mg five times a day for 10 days PO and was educated about getting the shingles vaccination.

The lifetime risks for incident CVD are higher in middle-aged females who are overweight or obese when compared to those with normal BMI. In a study involving a cohort of 140,835 female patients with a mean age of 58.7 years (standard deviation: 12.9 years), the risk ratios for CVD were 1.32 (95% CI: 1.24-1.40) for overweight women (BMI: 25.0-29.9 kg/m^2^) and 1.85 (95% CI: 1.72-1.99) for obese women (BMI: 30.0-39.9 kg/m^2^) compared to women of normal weight [13]. Higher BMI was significantly associated with incident HF among CVD patients [13]. Our patient’s BMI of 27.9 kg/m^2^ puts her at risk for developing CVD; she knows she has an increased BMI and follows a healthy diet and exercises regularly.

Lip et al. (2022), studying a large cohort of 4.3 million US patients with MI in relation to comorbidities, confirmed that comorbid diabetes and hypertension are risk factors leading to poor outcomes [14]. Our patient was educated about controlling her blood pressure and was advised to continue with lisinopril 20 mg daily to treat her primary hypertension. She is aware that she has elevated HbA1C levels and follows a healthy diet. In six months, she needs to repeat the HbA1C test as she has prediabetes.

RETRACTED

Our patient had been previously diagnosed with hypercholesterolemia, which was well controlled on 10 mg of atorvastatin daily. Since the patient was diagnosed with SMI, she was advised to increase her dose of atorvastatin from 10 to 80 mg daily. Atorvastatin is a high-intensity statin that is effective in the primary and secondary prevention of MI [15]. The intensive atorvastatin therapy (80 mg/day) versus the same dosage of simvastatin and low-dosage atorvastatin reduces the risk of nonfatal MI by 17-22% (p≤0.02). Atorvastatin versus usual care reduced the risk of nonfatal MI by 47-59% (p≤0.0002). Atorvastatin versus placebo, pravastatin, or simvastatin has been shown to reduce the risk of death or major cardiovascular events by 16-18% (p≤0.048) [15].

According to MIRKB, our patient is at risk of developing recurrent MI [7]. The patient is uninsured. The family practice for uninsured patients does not have the equipment to conduct a stress echocardiogram. As part of her continued care, she was referred to a cardiologist. The stress test should then be completed to assess further for CAD or arrhythmia. The 2014 Appropriate Use Criteria (AUC) guidelines focused on testing for CAD and summarized the evidence and provided recommendations for test selection [16]. The patient can exercise so that she can undergo a low-cost exercise-ECG test (treadmill-ECG). If the result of this test is abnormal, she should do the stress echo-exercise test or stress nuclear-exercise test [single photon emission computed tomography (SPECT) or positron emission tomography (PET)] [16]. If the result of this test is abnormal, she should undergo cardiac CT angiography (CTA) or cardiac catheterization (Cath) [16,17].

Results from these tests would allow the clinician to stratify the CVD state, and a combined approach should be applied appropriately. This includes counseling the patient on a healthy diet and employing regular cardiovascular-physical exercise and stress relief therapy. Medication prescription is often made, and follow-up with the provider is planned to control the dynamic results of such interventions. If tests reveal ischemia, appropriate pharmacotherapy of antiplatelet drugs, such as aspirin, and lipid-lowering drugs, such as statins, should be applied. Recent evidence supports the prescription of low doses of direct anticoagulants or a second antiplatelet agent for patients with a history of previous MI.

If a stress test detects an arrhythmia, the patient should be educated to avoid caffeine, alcohol, and tobacco and to manage her blood pressure, weight, and blood sugar levels [18]. If arrhythmia does not need any treatment, regular checkups should be recommended. If arrhythmia needs treatment, antiarrhythmic medications such as sodium channel blockers, beta-blockers, potassium channel blockers, nondihydropyridine calcium channel blockers, adenosine, or digoxin could be prescribed [18].

RETRACTED

## Conclusions

Our patient, who was following up on a recent shingles outbreak, mentioned experiencing skipped heartbeats and heart rate fluctuations and subsequently underwent an ECG, which led to a diagnosis of SMI in correlation with the patient's symptoms and risk factors. The tests other than ECG were not available at the family practice clinic. The patient was educated on MI symptoms, advised to call 911 if chest pain or SOB occurred, and referred for further consultation with a cardiologist. Based on other identified risk factors, including high BMI, prediabetes, primary hypertension, hypercholesterolemia, and HZ, the patient was advised to continue with lisinopril 20 mg daily, prescribed atorvastatin 80 mg daily, and was educated about maintaining a healthy diet, exercise, and receiving the shingles vaccination. Since the sensitivity and specificity of ECG alone are insufficient, the patient was referred to a cardiologist to undergo a stress test to assess further for CAD or arrhythmia. Further research is needed to devise and implement affordable screening methods for identifying SMI in family practice clinics.
